# Stereotactic Aspiration Acts as an Effective Treatment for Malignant Middle Cerebral Artery Infarction

**DOI:** 10.1155/2022/4373404

**Published:** 2022-04-16

**Authors:** Zhiyu Wang, Maogang Chen, Chong Wang, Jinbiao Luo, Shujie Sun, Xiangui Lu

**Affiliations:** ^1^Department of Neurosurgery, Xuhui Central Hospital, Zhongshan-Xuhui Hospital, Affiliated to Fudan University, Shanghai Clinical Center CAS, Shanghai 200031, China; ^2^Department of Neurosurgery, Jinling Hospital, School of Medicine, Nanjing University, Nanjing, Jiangsu 211299, China; ^3^Department of Emergency, The People's Hospital of Suzhou New District, Suzhou, Jiangsu 215129, China; ^4^Department of Neurosurgery, Guangzhou First People's Hospital, Guangzhou, Guangdong 510180, China

## Abstract

**Objective:**

This study seeks to explore the efficacy and prognosis of stereotactic aspiration for malignant middle cerebral artery infarction (mMCAI).

**Methods:**

A total of 50 mMCAI patients who were diagnosed and treated in our hospital from January 2018 to June 2020 were collected and then randomly divided into control group (decompressive craniectomy, *n* = 24) and study group (stereotactic aspiration, *n* = 26). After 1 and 6 months of treatment, the scores of the National Institutes of Health Stroke Scale (NIHSS), Glasgow Coma Scale (GCS), Barthel Index, and modified Rankin Scale (mRS) were used to evaluate the therapeutic effect. Additionally, the mortality and survival rates after treatment were recorded to compare the prognostic effect between the two groups.

**Results:**

One month after treatment, the GCS scores and Barthel Index score increased in both the control and study groups and were significantly higher in the study group. The follow-up results at 1 and 6 months after treatment showed that in comparison with the control group, stereotactic aspiration led to a higher survival rate and lower mortality rate; the latter had superior NIHSS score and mRS score and better prognosis.

**Conclusion:**

In comparison with decompressive craniectomy, stereotactic aspiration shows outstanding clinical efficacy and more advantages in the treatment of mMCAI. Therefore, stereotactic aspiration is more worthy of clinical application.

## 1. Introduction

Malignant middle cerebral artery infarction (mMCAI) is a special type of large hemispheric infarction [1]. Space-occupying cerebral edema progresses rapidly in the early stages of mMCAI, causing refractory intracranial hypertension and consequently rapid neurological deterioration and brain herniation within 24–72 h after onset [1]. Its mortality rate is still as high as 80% even after optimal conservative treatment [2], and survivors still have a severe disability [3]. Decompressive craniectomy (DC) is previously recognized as an effective means to significantly reduce intracranial pressure (ICP) in mMCAI patients, effectively prevent the expansion of infarcts, and therefore reduce mortality [4–7]. A meta-analysis by Das et al. [8] confirmed a low mortality rate but a high disability rate in patients with mMCAI after DC treatment compared to drug treatment. García-Feijoo et al. [9] also found that DC in patients with mMCAI leads to severe neurological sequelae, but the technique is still accepted by most patients in order to ensure their survival. Therefore, DC for mMCAI is still controversial within the medical community, and the treatment that is more minimally invasive and effective is required to be further explored.

At present, stereotactic aspiration is regarded as an emerging effective treatment for hypertensive intracerebral hemorrhage (HICH) by aspirating necrotic brain tissue [10, 11]. A case report study showed that stereotactic aspiration of necrotic brain tissue is an effective and safe method in patients over 60 years of age with mMCAI [12]. Stereotactic aspiration could reduce brain capacity by aspirating necrotic brain tissue [13]. The operation may minimize the release of toxic substances such as leukotrienes, interleukins, and platelet-activating factor from necrotic tissue which could reduce the damage and edema of surrounding normal brain tissue [14, 15]. In stereotactic aspiration of necrotic brain tissue, intraoperative bleeding is a major concern [12, 13]. Despite the fact that stereotactic aspiration of necrotic brain tissue reduced brain edema, the procedure alone did not always relieve ICP [12, 16]. Moreover, because of technical limitations and high cost, the operation is still limited to a small-scale retrospective study. There are no studies comparing the clinical efficacy of DC versus stereotactic aspiration for mMCAI. Therefore, we conducted a randomized controlled trial (RCT) to investigate the effectiveness and prognosis of DC and stereotactic aspiration therapy in patients with mMCAI.

## 2. Materials and Methods

### 2.1. Study Subjects

This study was a RCT. Fifty mMCAI patients who were diagnosed and treated in our hospital from January 2018 to June 2020 were collected and then randomly divided into control group (DC, *n* = 24) and study group (stereotactic aspiration, *n* = 26). Informed consent was obtained from all participants, and this study was approved by the Medical Ethics Committee of Shanghai Xuhui Central Hospital (2019-087-001).

Patient inclusion criteria were developed according to the surgical criteria of DC for mMCAI: [17] (1) clinical manifestations of complete hemiplegia, hemianesthesia, hemianopia, gaze disorder, and/or with higher neurological dysfunction (such as aphasia, a disorder of consciousness); (2) National Institutes of Health Stroke Scale (NIHSS) score ≥15 points; (3) LHI confirmed by cranial MRI or CT: 2/3 of the middle cerebral artery area with or without the involvement of ipsilateral anterior (and/or posterior) cerebral artery areas; (4) 24–48 h after onset; (5) preoperative CTA confirmed the occlusion of large vessels in the infarcted area.

Exclusion criteria were as follows: [18] (1) a history of stroke and severe sequelae; (2) acute infarction of both cerebral hemispheres; (3) having received intravenous thrombolysis and/or intra-arterial thrombolysis or mechanical thrombectomy; (4) hemorrhagic transformation and subsequently severe mass effect; (5) bilateral mydriasis and brainstem failure; (6) coagulation disorders. Patients who met the inclusion criteria were randomized to the control and study groups, with the consent of their families.

### 2.2. Surgical Methods

Before surgery, routine medication was given to control cerebral edema and the vital signs of patients were monitored, with open airway, indwelling catheter, gastrointestinal decompression, and deep venous catheterization. Patients were preoperatively given adequate sedation, analgesia, and antiemetic, along with control of blood pressure. Additionally, patients received conventional internal medical treatment for complications, nutritional support, or others.

The control group was treated with DC. After general anesthesia using endotracheal intubation, the patients were placed in the supine position. Standard large frontotemporoparietal DC was carried out. The cerebral dura mater was opened, and resection of the infarcted brain tissue was performed, not depending on the conditions of encephalocele [19]. The operative area was thoroughly hemostatic, and a drainage tube was placed at the flap.

The study group was preoperatively given intubation in the contralateral lateral ventricle to release 5–10 mL of cerebrospinal fluid and therefore to reduce the intracranial pressure. Then, patients received local anesthesia using lidocaine or general anesthesia with endotracheal intubation [20]. The following specific steps were undertaken: (1) according to the principle of stereotactic removal of hematoma [21], the head stereoscopic drawing method was used to draw the horizontal, coronal, and sagittal planes of the cranial surface where the puncture point and the puncture direction line are located on the head. (2) Determine the puncture target (usually 1–3), the puncture path, and the depth of puncture according to the largest dimension of the infarct area by referring to the CT positioning of the patient's head. (3) After determining the puncture point and sterilizing with routine anesthesia, a bone hole with a diameter of about 7 mm was drilled along the puncture direction by using a cranial drilling tool. Then, after the drilling resistance was felt to disappear, the directional drilling tool was removed. Next, the concave cranial drill was adopted for cleaning the bone debris in the bone hole, followed by placement of the keyhole device. (4) The dura mater was punctured with a meningeal puncture needle through the keyhole device, and then a three-level smooth probe was used for slow and progressive expansion along the keyhole device to establish a prechannel. (5) A soft tube was placed into the infarcted tissue, followed by aspiration of necrotic brain tissue with a 20 mL syringe. After aspiration, 500 mL of normal saline were used to rinse until no active bleeding. Then, the drainage bag was connected to continue open drainage. The occupancy effect of cranial CT and cranial hypertension was observed 2–5 d after surgery. Generally, after drainage for 5–7 days, the clinical symptoms were improved and head CT was reexamined.

### 2.3. Barthel Index

The total score is 100, including 10 items: feeding, bathing, grooming, dressing, bowels, bladder, toilet use, transfers (bed to chair and back), mobility (on level surfaces), and stairs. The higher the score, the higher the quality of daily life.

### 2.4. National Institutes of Health Stroke Scale

National Institutes of Health Stroke Scale (NIHSS) includes the following items: level of consciousness, best gaze, visual, facial palsy, motor arm, motor leg, limb ataxia, sensory, best language, dysarthria, and extinction and inattention. The specific scoring criteria can be found in the appendix of the study by Chen [22]. The higher the score, the more serious the nerve injury.

### 2.5. Glasgow Coma Scale

Glasgow Coma Scale (GCS) includes 3 kinds of responses: eye-opening response, verbal response, and motor response. Eye-opening response is scored as 4 (spontaneous), 3 (to verbal stimuli), 2 (to pain), and 1 (no response). A verbal response is scored as 5 (oriented), 4 (confused conversation), 3 (inappropriate words), 2 (incomprehensible speech), and 1 (no response). Motor response is scored as 6 (obey command), 5 (purposeful movement to painful stimulus), 4 (withdraws to pain), 3 (decorticate posturing), 2 (decerebrate posturing), and 1 (no response) [23]. A high GCS score indicates that the patient's consciousness is weak.

### 2.6. Modified Rankin Scale

The total score of modified Rankin Scale (mRS) is 0–6, and the specific score description is as follows: 0, no symptoms at all; 1, slight symptoms: able to complete all daily life and work; 2, slight disability: unable to complete all activities, but no need for assistance to own daily life; 3, moderate disability: need some help, but can walk independently; 4, moderately severe disability: unable to walk independently and unable to attend to own daily life; 5, severe disability: bedridden, incontinence, and daily life completely dependent on others [24]. The lower the score, the less the degree of nerve injury.

### 2.7. Statistical Analysis

With SPSS 21.0 for statistical analysis, the measurement data were analyzed by two-sample *t*-test and expressed as mean ± standard deviation (SD). By contrast, enumeration data were expressed by *n* (%) and analyzed by the chi-square test. A significant difference was suggested if *P* < 0.05.

## 3. Results

### 3.1. Baseline Data

A total of 50 patients were included, including 27 males and 23 females, with an average age of 55 years (40–69 years) and an infarction volume ranging from 142 to 175 ml. The study subjects included 26 cases with a previous history of hypertension, 21 with diabetes, and 25 with atrial fibrillation. Their NIHSS scores ranged from 15 to 21. No significant differences were identified between the two groups in gender, age, infarction diameter, comorbidities, and NIHSS score (*P* > 0.05), suggesting comparability (Table 1).

### 3.2. CT Images

Preoperative CT in one patient revealed a large cerebral infarction in the left middle cerebral artery territory, accompanied by severe cerebral edema and marked midline shift (Figure 1(a)). On the second day after stereotactic aspiration, CT examination observed the drainage tube placed into the infarct lesion through the frontal and temporal lobes, respectively, and partially reduced midline shift (Figure 1(b)). The CT image at the 8th week after surgery showed encephalomalacia foci in the infarcted area, complete reduction of midline shifts, and relief of lateral ventricle compression (the drainage tube had been removed on the 5th day after surgery) (Figure 1(c)).

### 3.3. Comparison of Daily Living in Patients with mMCAI

We compared the two groups of patients by GCS score and Barthel Index score for daily living ability. Before treatment, there was no significant difference in GCS score and Barthel Index score between the control group and the study group (*P* > 0.05), and the two groups were comparable. The GCS score and Barthel Index score of the two groups after 1 month of treatment were significantly higher than those before surgery (*P* < 0.05). In comparison with the control group, patients in the study group achieved significantly higher GCS and Barthel Index scores at 1 month after stereotactic aspiration (Table 2).

### 3.4. Comparison of Neurological Function in Patients with mMCAI

The degree of neurological deficit and neurological recovery was evaluated by the NIHSS and mRS scores, respectively. The NIHSS scores and mRS scores of the two groups before treatment were not significantly different (*P* > 0.05), suggesting that the preoperative neurological functions of the two groups were comparable. The NIHSS score and mRS score of the two groups after 1 and 6 months of treatment were significantly lower than those before surgery. Furthermore, in comparison with the control group, the study group achieved significantly lower NIHSS and mRS scores at 1 and 6 months after stereotactic aspiration (Table 3).

### 3.5. Comparison of Prognosis in Patients with mMCAI

Survival and mortality and sequelae of the two groups were counted for comparing the prognostic effects of the two treatments. As shown in Table 4, the survival rate and the recovery rate were significantly higher in the study group compared with the control group (53.85% vs. 16.67%), and only one patient died with a significantly lower mortality rate (*P* < 0.05). We further evaluated the side effect rates (including disability and vegetative state) of both treatment modalities and found that the control group had a significantly higher disability and vegetative state rate compared to the study group, suggesting that stereotactic aspiration has a superior outcome and prognosis.

## 4. Discussion

mMCAI, as the main fatal cerebrovascular disease, is harmful to human health, thus requiring treatment with good therapeutic effect and good prognosis. In recent years, mMCAI has been explored in the fields of pathogenesis, clinical features, early diagnosis, treatment strategies, and prognostic management [2, 17, 25, 26]. Although conservative internal medical treatment is mostly adopted for mMCAI in clinical practice, the timely surgical intervention also shows a significant effect on improving the prognosis of some patients [27]. Stereotactic aspiration therapy, an emerging method with easy operation, greatly shortens the time required for surgery and strives for more valuable time for HICH patients. Additionally, stereotactic aspiration for HICH causes less trauma and therefore contributes to the postoperative recovery of patients; it also puts lower technical requirements and therefore is beneficial to promotion in primary hospitals [28, 29]. However, its role in mMCAI is still not fully understood, so stereotactic aspiration therapy should still be studied in depth [30].

In this study, we compared the efficacy of DC and stereotactic aspiration therapy in patients with mMCAI. The results showed that the GCS scores and Barthel Index were significantly higher in patients with mMCAI after stereotactic aspiration therapy compared to DC, suggesting a significant improvement in patients' ability to perform daily living after surgery. In addition, after 6 months of treatment, patients in the stereotactic aspiration therapy group had significantly lower NIHSS scores and mRS scores compared to the DC group. This is similar to the findings of Kilic et al. [31]. The study showed that mMCAI patients generally exhibit lower GCS scores as well as higher mRS scores in the DC group compared with patients in the conservative treatment group [32]. This suggests that stereotactic aspiration therapy is more effective than DC for mMCAI. In addition, patients in the stereotactic aspiration therapy group had better recovery of consciousness, significantly better survival, significantly lower mortality, and better prognosis than those in the DC group. Other studies have shown that early stereotactic aspiration of necrotic brain tissue within 24 to 48 h after onset is safe and effective for mMCAI patients aged over 60 years, which can reduce mortality and improve long-term prognosis [20]. This result is consistent with ours. However, this study was conducted on patients with mMCAI over 60 years of age. Kilic et al. [31] also indicated that patients with mMCAI over 60 years of age still showed lower GCS scores and higher mRS scores after DC treatment within 24 h. In contrast, the age level of patients was not divided for the study, whose main limitation was the small sample size. Therefore, we need to further expand the clinical sample for mMCAI treatment study.

## 5. Conclusion

In summary, in comparison with DC, stereotactic aspiration shows better efficacy and prognosis in the treatment of mMCAI. It is suggested that stereotactic aspiration is a feasible and effective treatment for mMCAI in clinical practice.

## Figures and Tables

**Figure 1:** Preoperative and postoperative brain CT images of a patient. (a) Preoperative CT image: A, infarct in the left middle cerebral artery territory; B, less lateral ventricle compression on the infarct side. (b) CT image 2 days after surgery: A, drainage tube placed into the infarct focus through the frontal part; B, drainage tube placed into the infarct focus through the temporal part. (c) CT image 8 weeks after surgery: A, encephalomalacia foci in the infarct area; B, complete reduction of midline shifts and complete relief of lateral ventricle compression.

**Table 1:** Comparison of clinical characteristics of patients before surgery.

		Control group (*n* = 24)	Study group (*n* = 26)	*χ* 2/*F*	*P* value
Gender (male/female)		13/11	14/12	0.297	>0.05
Age (years)		158.58 ± 8.15	161.15 ± 7.60	0.284	>0.05
Infarction volume (ml)		92.06 ± 6.93	93.03 ± 3.62	0.048	>0.05
Comorbidity	Hypertension	12	14	0.074	>0.05
	Diabetes	10	11	0.093	>0.05
	Atrial fibrillation	13	12	0.125	>0.05
NIHSS score		18.38 ± 3.58	19.34 ± 2.92	0.198	>0.05

Values are mean ± SD or numbers.

**Table 2:** Comparison of GCS and Barthel Index scores in the two groups before and after treatment.

		Control group (*n* = 24)	Study group (*n* = 26)	*t* value	*P* value
GCS scores	Before treatment	8.22 ± 1.27	8.29 ± 1.44	0.192	>0.05
	1 month after treatment	10.46 ± 1.92^*∗*^	13.40 ± 1.65^*∗*Δ^	6.255	<0.05

Barthel Index	Before treatment	35.06 ± 4.85	35.69 ± 4.55	0.008	>0.05
	1 month after treatment	43.99 ± 7.91^*∗*^	60.29 ± 9.00^*∗*^^∆^	6.299	<0.05

Values are mean ± SD. ^*∗*^*P* < 0.05 vs. before treatment; Δ*P* < 0.05 vs. control group (1 month after treatment).

**Table 3:** Comparison of NIHSS score and mRS score in the two groups before and after treatment.

Group		Control group (*n* = 24)	Study group (*n* = 26)	*t* value	*P* value
NIHSS score	Before treatment	17.17 ± 6.31	18.34 ± 6.24	0.147	>0.05
	1 month after treatment	15.70 ± 5.34^*∗*^	11.26 ± 4.18^*∗*Δ^	2.417	<0.05
	6 months after treatment	11.44 ± 3.80^*∗*^	9.05 ± 2.79^*∗*Δ^	4.068	<0.05

mRS score	Before treatment	4.14 ± 0.46	4.57 ± 0.86	0.046	>0.05
	1 month after treatment	3.26 ± 0.16^*∗*^	2.25 ± 0.29^*∗*Δ^	17.594	<0.05
	6 months after treatment	1.01 ± 0.09^*∗*^	0.11 ± 0.03^*∗*Δ^	53.472	<0.05

Values are mean ± SD. ^*∗*^*P* < 0.05 vs. before treatment; Δ*P* < 0.05 vs. control group (1 or 6 months after treatment).

**Table 4:** Comparison of prognosis in the two groups.

	Control group (*n* = 24)	Study group (*n* = 26)	*P* value
Recovered	4 (16.67)	14 (53.85)	<0.05
Slight disability	7 (29.17)	4 (15.38)	<0.05
Moderate disability	5 (20.83)	3 (11.54)	<0.05
Severe disability	3 (12.50)	2 (7.69)	<0.05
Vegetative state	3 (12.50)	2 (7.69)	<0.05
Death	2 (8.33)	1 (3.85)	<0.05

Values are *n* (%).

## Data Availability

The data used to support the findings of this study are available from the corresponding author upon request.
